The article "Curcumin-Chitosan Nanocomposite Formulation Containing Pongamia pinnata-Mediated Silver Nanoparticles, Wound Pathogen Control, and Anti-Inflammatory Potential" was retracted in 2024. Reasons: signs of a paper mill; compromised peer review; unreliable results or conclusions.

# Curcumin-Chitosan Nanocomposite Formulation Containing *Pongamia pinnata*-Mediated Silver Nanoparticles, Wound Pathogen Control, and Anti-Inflammatory Potential

**DOI:** 10.1155/2021/3091587

**Published:** 2021-12-23

**Authors:** Rajeshkumar Shanmugam, Rajaduraipandian Subramaniam, Sabeena Gabrial Kathirason, Daoud Ali, Sri Renukadevi Balusamy, Annadurai Gurusamy, Kalirajan Arunachalam, Hanen Sellami

**Affiliations:** ^1^Department of Pharmacology, Saveetha Dental College and Hospital, SIMATS, Chennai 600077, India; ^2^Research Department of Chemistry, Sri Paramakalyani College, Sri Paramakalyani Centre of Excellence in Environmental Sciences, Manonmaniam Sundaranar University, Alwarkurichi, 627412, India; ^3^Department of Zoology, College of Science, King Saud University, Riyadh, P.O. Box 2455, 11451, Saudi Arabia; ^4^Department of Food Science and Biotechnology, Sejong University, Gwangjin-gu, Seoul 05006, Republic of Korea; ^5^Department of Science and Mathematics, School of Science, Engineering and Technology, Mulungushi University, Kabwe 80415, Zambia; ^6^Laboratory of Treatment and Valorization of Water Rejects (LTVRH), Water Researches and Technologies Center (CERTE), Borj Cedria Technopark, University of Carthage, 8020 Soliman, Tunisia

## Abstract

**Background:**

Because of its diverse range of use in several ethics of diagnosis and care of multiple diseases, nanotechnology has seen remarkable growth and has become a key component of medical sciences. In recent years, there has been rapid advancement in medicine and biomaterials. Nanomedicine aids in illness prevention, diagnosis, monitoring, and treatment.

**Aim:**

The purpose of this work is to evaluate the antibacterial, anti-inflammatory, and cytotoxic capabilities of green produced silver nanoparticle with the addition of curcumin-assisted chitosan nanocomposite (SCCN) against wound pathogenic as reducing agents.

**Materials and Methods:**

The plant extract of *Pongamia pinnata*, silver nanoparticles, and its based curcumin nanoformulations was studied in this study utilizing UV visible spectrophotometer, selected area electron diffraction (SAED), and TEM. Anti-inflammatory, antimicrobial, and cytotoxic tests were performed on silver nanoparticles with the addition of curcumin-assisted chitosan nanocomposite (SCCN). Furthermore, these produced nanocomposites were coated on clinical silk and tested for antibacterial activity.

**Results:**

The produced silver nanoparticle with the addition of curcumin-assisted chitosan nanocomposite (SCCN) has significant antibacterial activities against *Pseudomonas aeruginosa and staphylococcus aureus*. They are as well as possess anti-inflammatory activity and furthermore prove to be biocompatible.

The article "Curcumin-Chitosan Nanocomposite Formulation Containing Pongamia pinnata-Mediated Silver Nanoparticles, Wound Pathogen Control, and Anti-Inflammatory Potential" was retracted in 2024. Reasons: signs of a paper mill; compromised peer review; unreliable results or conclusions.

**Conclusion:**

This advancement in the field of biomaterials, which means nanocomposite, not only helps to reduce the harmful effects of pathogenic organisms while representing an environmentally benign material but it also shows to be a material with zero danger to humans and the environment.

## 1. Introduction

Nanotechnology has grown tremendously in the last decade, becoming an essential component of medical sciences as a result of its broad variety of applications in many concepts of illness investigation and therapy [1]. Recently, the literature has demonstrated a possible function for metal nanoparticles as antibacterial agents. However, the functional characteristics of metal nanoparticles may be improved to round out the green production technique. Due to its pharmacological medication and biodistribution activities, researchers are now working on nanobased pharmaceuticals, for example, they offer a platform intended at operative delivery of drug molecules. The use of nanobased pharmaceuticals to accomplish conservative techniques comparable to their physical and chemical ways has been proven to be hazardous to the environment due to the use of noxious chemicals or the use of excessive temperature or pressure circumstances. Researchers are focusing more on biological approaches that include plant and its components and microorganisms comparable to fungus, algae, and bacteria, in order to complete the nontoxic, environmentally friendly method utilized for nanoparticle production [2–7].

Green synthesis is a preferred way for concluding other processes due to the movability of created nanomaterials and repeatability [8]. From algae [9], actinomycetes [10], sugar [11], biodegradable polymers (chitosan) [12], bacteria [13], and plants [14], nanoparticles have been efficiently manufactured. Plant-mediated synthesis, in the middle of the abovementioned approaches, is measured faster and requires less tuning [15].

Curcumin's antioxidant, anti-inflammatory, antitumor, and antimicrobial activities remain powerful [16]. They offer several therapeutic properties with a higher safety profile, but administration is complicated. Its disadvantages include poor bioavailability, rapid metabolism, and inadequate absorption [17]. Huge amounts must be thought to have reached the significant concentration. To address these issues, nanoparticle-based drug delivery techniques are the best option for expanding curcumin's medicinal uses [18]. Because these materials have the ability to enter tissues and organs, translocate to other cells, penetrate cells, and be withdrawn from the gateway of admission to the body [19], cultivating their bioavailability is conceivable for aiding in the treatment of a variety of oral diseases.

The article "Curcumin-Chitosan Nanocomposite Formulation Containing Pongamia pinnata-Mediated Silver Nanoparticles, Wound Pathogen Control, and Anti-Inflammatory Potential" was retracted in 2024. Reasons: signs of a paper mill; compromised peer review; unreliable results or conclusions.

*Pongamia pinnata* is a crude medicine used to treat skin problems, ulcers, tumours, and piles [20, 21]. The *Pongamia pinnata* root is a surgical tool used to treat teeth, ulcers, and gum disease. Furthermore, it is reused in skin illnesses and vaginal wounds [22]. Tribal tribes in modern day southern India employed this herb to cure wounds in the trendy Ayurvedic therapeutic method. *Pongamia pinnata* stem bark is diversified with the wide-ranging plant to be put topically on exaggerated regions to treat wounds; however, the combination of *Pongamia pinnata* oil is also useful to heal wounds [23].

Silver nanoparticles (Ag NPs) were organized using a variety of processes, including physical, biological, chemical, and green methods [24]. Ag NPs have high antimicrobial capabilities and may be employed effectively against multidrug-resistant pathogens [25]. Ag NPs are particularly advantageous due to their high specific poisonousness towards bacteria and low toxicity towards humans.

In this work, green produced silver nanoparticles with the addition of curcumin-assisted chitosan nanocomposite (SCCN) were used to combat wound pathogenicity and were analyzed utilizing various spectroscopic analyses such as UV, TEM, and SAED. Based on antibacterial, cytotoxicity, and anti-inflammatory properties, this nanoparticle-based nanocomposite was the optimum technique for large-scale manufacture.

## 2. Materials and Methods

### 2.1. Materials

Sigma–Aldrich supplies all the chemicals, and we used these chemicals for fashionable experiments. Curcumin, silver nitrate, chitosan, and bacterial media were commercially purchased from Hi Media, Mumbai. With the assistance of double distilled water, the entire research experiment was carried out.

### 2.2. Preparation of Plant Extract and Silver Nanoparticle Synthesis

*Pongamia pinnata* known as a medicinal herb was properly cleaned with tap water and cut into little pieces to dry in the shade for 3-4 days. The shade dried leaf fragments were then ground into a fine powder. Following that, 0.7 g of finely ground *Pongamia pinnata* powder was added to 70 mL of distilled water. For 15 minutes, the mixture was kept warm in an 80°C heating mantle. The hot mixture was previously filtered via Whatman No. 1 filter paper. The filtered *Pongamia pinnata* extract was placed in a refrigerator to produce nanoparticles. In 500 mL Erlenmeyer flasks, a 2 mM aqueous AgNO_3_ solution was prepared. An orbital shaker was used to protect the flasks containing the extract. The colour changes in the reaction mixture were tested continuously over a long period using a double beam UV-visible spectrophotometer next to different wavelength sections ranging from 350 to 550 nm. The green produced Ag NPs were centrifuged for 15 minutes at 10,000 rpm before being collected.

The article "Curcumin-Chitosan Nanocomposite Formulation Containing Pongamia pinnata-Mediated Silver Nanoparticles, Wound Pathogen Control, and Anti-Inflammatory Potential" was retracted in 2024. Reasons: signs of a paper mill; compromised peer review; unreliable results or conclusions.

### 2.3. Preparation of Nanoformulation and Nanocomposite

For the preparation of the nanocomposite, 100 mg of curcumin was mixed with 5 mL of DMSO, and the solution was mixed with Ag NPs. For the preparation of the nanocomposite, 25 mL of chitosan was mixed with Ag NPs with curcumin formulation and kept in magnetic stirrer for 24 hours. To eliminate any suspended particles, nanoformulation and nanocomposite were filtered using Whatman No. 1 filter paper. Finally, a clean filtrate was produced and employed for nanoformulation and the fabrication of nanocomposite materials.

### 2.4. Anti-Inflammatory Activity

Chemicals required for anti-inflammatory action, such as bovine serum albumin, 1 N HCl, phosphate buffer (pH 6.3), and then the following four solutions, were utilized. The first test solution (0.5 mL) contains 0.5 mL of bovine serum albumin and 0.06 mL of test resolution in many attentions, and the pH will be adjusted to 6.3 using a tiny quantity of 1 N HCl. The samples were heated at 60°C for 5 minutes after being incubated at 37°C for 30 minutes. After cooling, 3 mL of phosphate buffer (pH 6.3) was added to the sample, followed by 0.5 mL of test control solution (0.5 mL) containing 0.5 mL of bovine serum albumin and 0.06 mL of distilled water, and then the pH was adjusted to 6.3 using a pH meter by means of small amount of 1 N HCl. The samples were heated at 60°C for 5 minutes after being incubated at 37°C for 30 minutes. After cooling, 3 mL of phosphate buffer was added to the sample (pH 6.3). Third, a product control solution (0.5 mL) was made out of 0.5 mL of distilled water and 0.06 mL of test solution in varied concentrations, and the pH was adjusted to 6.3 using a little quantity of 1 N HCl. The samples were heated at 60°C for 5 minutes after being incubated at 37°C for 30 minutes. After cooling, 3 mL of phosphate buffer was added to the sample (pH 6.3). Finally, the fourth standard solution (0.5 mL) was made up of 0.5 mL of bovine serum albumin and 0.06 mL of diclofenac sodium solution at various concentrations, and the pH was adjusted to 6.3 by means of small amount of 1 N HCl. The samples were incubated at 37°C for 30 minutes and heated at 60°C for 5 minutes. After subsequently freezing, 3 mL of phosphate buffer (pH 6.3) was added to the sample. The percentage reserve of protein denaturation was calculated as follows [26].

(1) $$\begin{array}{c} \text{Percentage inhibiton}=\frac{{\text{Abs}}_{\text{control}}-{\text{Abs}}_{\text{sample}}\;}{{\text{Abs}}_{\text{control}}}\times 100\; \end{array}$$

The control signifies 100% protein denaturation. The result will be associated with diclofenac sodium treated samples.

The article "Curcumin-Chitosan Nanocomposite Formulation Containing Pongamia pinnata-Mediated Silver Nanoparticles, Wound Pathogen Control, and Anti-Inflammatory Potential" was retracted in 2024. Reasons: signs of a paper mill; compromised peer review; unreliable results or conclusions.

### 2.5. Antimicrobial Activity Using Agar Well Diffusion Assay

The agar well diffusion technique was used to determine the initial antibacterial activity of silver nanoparticles with the addition of curcumin-assisted chitosan nanocomposite (SCCN) against oral pathogenic gram-positive and gram-negative bacteria [27]. The changing attentions of manufactured nanoparticles were tested against harmful microorganisms such as *Staphylococcus aureus* and *Pseudomonas aeruginosa*. In Muller-Hinton agar plates, silver nanoparticles with curcumin-assisted chitosan nanocomposite (SCCN) were concentrated to 100, 200, 300, 400, 500, and 1000 *μ*g/mL. The plates were incubated for 24 hours at 37°C, and the implications were noted by evaluating the diameter of the zone of inhibition in millimeters.

### 2.6. Growth Kinetic Assay

The effect of silver nanoparticle with the addition of curcumin-assisted chitosan nanocomposite (SCCN) on the growth kinetics of *Pseudomonas aeruginosa and staphylococcus aureus* separates was observed by optical density quantities [28]. Double dilution of silver nanoparticle with the addition of curcumin assisted chitosan nanocomposite (SCCN) extending from 20 *μ*g/mL to 320 *μ*g/mL was finished in a sterile 96-well microtiter fashionable plate in the nutrient broth. Ten *μ*L of the overnight grown culture (∼10^6^ CFU/mL) was immunized in every well covering variable concentrations of silver nanoparticle with the addition of curcumin-assisted chitosan nanocomposite (SCCN). Wells comprising only media were occupied as the control group, and every single concentration was achieved in three imitates. All unprocessed and conserved fashionable sample plates were incubated for 20 hours at 37°C. The OD_620nm_ was documented at intervals of 2 hours consuming a microplate reader (Thermo Scientific Multiskan EX, REF 51118170, China). The most common of three imitates was used to create the growth curve of each culture on the side of each and every concentration of nanoparticles. The growth inhibition ratio was estimated using the formula below:

(2) $$\begin{array}{c} \text{Growth inhibition percentage}=\frac{\text{Initial absorbance}-\text{Final absorbance}}{\text{Initial absorbance}}\times 100 \end{array}$$

### 2.7. Cytotoxicity Assay

The cytotoxicity of silver nanoparticle with the addition of curcumin-assisted chitosan nanocomposite (SCCN) was measured in the direction of human colon carcinoma cell line (HCA-7) finished of methyl thiazolyl tetrazolium (MTT) assay. The 2 × 10^4^ cells per well were sowed in a 100 mL intermediate in 96-well plates and were incubated overnight. Following incubation, the cells were maintained using varying concentrations of silver nanoparticles with the addition of curcumin-assisted chitosan nanocomposite (SCCN) (50-800 *μ*g/mL) and incubated for 24 hours. The plate was rinsed with PBS before adding 100 *μ*L of freshly prepared MTT solution (50 *μ*g/mL) via medium onto a 96-well plate and incubating it for 3–5 hours. Following the removal of MTT solution, 200 *μ*L of DMSO solution was added to the well, and the absorbance was measured at 570 nm. The experiment was completed in triplicates. The calculation was

(3) $$\begin{array}{c} \%\text{Inhibition}=\frac{\text{Absorbance of control}-\text{Absorbance of test sample}}{\text{Absorbance of the control}}\times 100 \end{array}$$

The important value of IC_50_ was considered by plotting a graph of absorption of silver nanoparticle with the addition of curcumin assisted chitosan nanocomposite (SCCN) using standard.

The article "Curcumin-Chitosan Nanocomposite Formulation Containing Pongamia pinnata-Mediated Silver Nanoparticles, Wound Pathogen Control, and Anti-Inflammatory Potential" was retracted in 2024. Reasons: signs of a paper mill; compromised peer review; unreliable results or conclusions.

### 2.8. Characterization

The UV-visible spectra of Ag NPs, Chitosan, and silver nanoparticles with the addition of curcumin-assisted chitosan nanocomposite (SCCN) with water as a blank were obtained using a Shimadzu UV-1800 spectrophotometer. TEM was used to determine the shape and size of the produced nanoparticles. To precisely estimate the size of nanoparticles, transmission electron microscopy was used. The sonicated sample was put onto a carbon-coated copper grid and allowed to dry overnight in a vacuum before being submitted to transmission electron microscopy and selected area electron diffraction (SAED) (FEI-TECNAI G220 TWIN).

## 3. Results and Discussion

### 3.1. Ultraviolet Spectroscopy

The UV image of Ag NPs, chitosan, and silver nanoparticles with the addition of curcumin-assisted chitosan nanocomposite (SCCN) is shown in Figure 1. UV-Vis spectroscopy was used to examine the creation of silver nanoparticles with the addition of curcumin-assisted chitosan nanocomposite (SCCN). Curcumin and chitosan both operate as reducing and stabilizing agents in the synthesis of Ag NPs in our work. To determine the best chitosan composition for the creation of Ag NPs, moderate conditions are used to prevent the use of reducing agents. The scanning of the solution with Ag NPs using ultraviolet-visible spectroscopy revealed an absorption peak at about 450 nm, which preliminarily confirmed Ag NP synthesis. The strength of the surface plasmon resonance absorption peak corresponding to Ag NPs has steadily grown (2.15 to 2.75) with a minor change in the peak's wavelength as the concentration of has increased (398 to 452 nm). The presence of a surface plasmon resonance absorption peak from 398 to 452 nm implies the development of smaller Ag NPs with a limited size distribution. The ultraviolet-visible region of silver nanoparticles with curcumin-assisted chitosan nanocomposite (SCCN) solution demonstrated a peak of absorbance at about 350 nm [29]. The ability to reduce as well as stabilize the produced nanoparticles improves of chitosan concentration due to the presence more number of reducible groups [30]. The solution containing chitosan has at 330 nm that is weak peak compared to other compositions. This indicates that the presence of curcumin and chitosan influences the reduction as well as the stabilization process of Ag NPs in the UV spectra.

The article "Curcumin-Chitosan Nanocomposite Formulation Containing Pongamia pinnata-Mediated Silver Nanoparticles, Wound Pathogen Control, and Anti-Inflammatory Potential" was retracted in 2024. Reasons: signs of a paper mill; compromised peer review; unreliable results or conclusions.

### 3.2. Selected Area (Electron) Diffraction

Selected area electron diffraction patterns (SAED) documented on the sections are presented in Figure 2. The observed Debye-Scherer rings are totally surrounded, representing the silver nanoparticle with the addition of curcumin-assisted chitosan nanocomposite (SCCN) nanostructure is decidedly crystalline nature. Selected area electron diffraction (SAED) through different amplifications confirmed the spherical crystalline nature of silver nanoparticle with the addition of curcumin assisted chitosan nanocomposite [31]. The ring modificationfrom continious to scattered based on the size of the nanoparticles. If the grains trendy the sample are focused on a favored direction, the SAED configuration shows that numerous rings are incomplete. If the sample is shapeless, diffuse rings will be achieved; although, crystalline samples will result in optimistic spots [32–37] and if the sample is delivered an overview of the SAED configuration of silver nanoparticle with the addition of curcumin-assisted chitosan nanocomposite (SCCN). Moreover, the framework fringe spacing established the face-centered cubic (fcc) nature of the silver nanoparticle with the addition of curcumin-assisted chitosan nanocomposite (SCCN) [38]. The results are arrangement with in the report by Quester et al. [39].

### 3.3. Transmission Electron Microscopy

The arrangement of the Ag NPs synthesized by using the plant extract *Pongamia pinnata* as green reducing agents is typically spherical in shape. The morphology of the Ag NPs were extremely adjustable with size range of 5 nm. In this study, TEM images obviously designated shape and size of the nanoparticle were practically alike with earlier study characterization [6, 40].  Figure 3 shows the transmission electron micrograph of Ag NPs and silver nanoparticle with the addition of curcumin assisted chitosan nanocomposite (SCCN). TEM images obviously demonstrated the diverse size range (200 nm) of Ag NPs and silver nanoparticle with the addition of curcumin-assisted chitosan nanocomposite (SCCN). Additionally, the transmission electron micrograph exposed that the greatest of the particles were spherical in shape along with few nanoparticles having anisotropic morphology. Few particles were also originate to form small aggregates, which possibly will be due to agglomeration or indecorous capping. The differences in shape and size of the nanoparticles and nanocomposite synthesized through green synthesis attitudes consumed similarly keep on recognized earlier [41, 42].

The article "Curcumin-Chitosan Nanocomposite Formulation Containing Pongamia pinnata-Mediated Silver Nanoparticles, Wound Pathogen Control, and Anti-Inflammatory Potential" was retracted in 2024. Reasons: signs of a paper mill; compromised peer review; unreliable results or conclusions.

### 3.4. Anti-Inflammatory Activity

The green mediated synthesis Ag NPs, silver nanoparticle with the addition of curcumin assisted chitosan nanocomposite (SCCN) shows analogous anti-inflammatory activity with standard dichlofenac sodium which is a chemical analgesic at different concentration (Figure 3). The green mediated synthesis Ag NPs, silver nanoparticle with the addition of curcumin-assisted chitosan nanocomposite (SCCN) can act as a powerful anti-inflammatory drug was shown in Figures 4 and 5. The in vitro bioassay results of anti-inflammatory effect of Ag NPs and silver nanoparticle with the addition of curcumin-assisted chitosan nanocomposite (SCCN) assessed that help reduce inflammation. The maximum inhibition on Ag NPs by *Pongamia pinnata* was found by 33% at 100 *μ*g/mL, 59% at 200 *μ*g/mL, 71% at 300 *μ*g/mL, 78% at 400 *μ*g/mL, and 81% at 500 *μ*g/mL, respectively. The concentration beyond 500 *μ*g/mL was found to be inhibitory more than 81% of the bacteria, and then the maximum inhibition on curcumin and chitosan was found to be 40% and 32% at 100 *μ*g/mL, 58% and 55% at 200 *μ*g/mL, 70% and 65% at 300 *μ*g/mL, 75% and 65% at 400 *μ*g/mL, and 80% and 74% at 500 *μ*g/mL in equal concentration, respectively. Silver nanoparticle with the addition of curcumin-assisted chitosan nanocomposite (SCCN) maximum inhibition percentage obtained was 45%, 60%, 68%, 75%, and 80% at a concentration of 100 *μ*g/mL, 200 *μ*g/mL, 300 *μ*g/mL, 400 *μ*g/mL, and 500 *μ*g/mL. When the concentration enlarged, the inhibition level of sample always increased.

### 3.5. Cytotoxicity Assay

Figure 6 shows the cytotoxic effect of nanoparticles and nanocomposites using brine shrimp lethality assay. The cytotoxic effect refers to a substance or process that results in cell damage. In this cytotoxic effect, control is stable for percentage calculation. The concentration level of 50 *μ*g/mL of Ag NPs represents 15%; at the same time, the concentration at 800 *μ*g/mL of Ag NPs represents 80%. When the concentration level increases, similarly percentage level also increased. The above graph shows that the Ag NPs, curcumin, and chitosan cytotoxic effects are separately demonstrated. The silver nanoparticle with the addition of curcumin-assisted chitosan nanocomposite (SCCN) was also revealed, and the concentration of 200 *μ*g/mL and 400 *μ*g/mL shows equal level of contribution in this cytotoxic effect at 30% of live Nauplii.

The article "Curcumin-Chitosan Nanocomposite Formulation Containing Pongamia pinnata-Mediated Silver Nanoparticles, Wound Pathogen Control, and Anti-Inflammatory Potential" was retracted in 2024. Reasons: signs of a paper mill; compromised peer review; unreliable results or conclusions.

### 3.6. Antibacterial Activity

The antimicrobial activity of silver nanoparticle with the addition of curcumin-assisted chitosan nanocomposite (SCCN) was investigated against *Pseudomonas aeruginosa* and *Staphylococcus aureus* using the agar well diffusion assay that revealed minimum inhibitory concentrations at various concentrations. The antimicrobial activity increases as well as increase in silver nanoparticle with the addition of curcumin-assisted chitosan nanocomposite (SCCN) concentration. The zones of minimum inhibition (mm) about each well comprising silver nanoparticle with addition of curcumin-based chitosan nanocomposite (SCCN) solution are signified in Figure 7. The antibacterial activity of silver nanoparticle with addition of curcumin-based chitosan nanocomposite (SCCN) against *Pseudomonas aeruginosa* was the highest by the range of 1000 *μ*L through zone of inhibition determining 18.5 mm while *Staphylococcus aureus* exposed zone of inhibition determining 16 mm, respectively. The improved antibacterial activity of silver nanoparticle with addition of curcumin-based chitosan nanocomposite (SCCN) solution was attributed to their large surface area that arrange for more surface interaction with microorganisms [43]. The mechanism of achievement of the antibacterial activity of Ag NPs is aggressive the respiratory chain and cell division that eventually information to cell death. The silver nanoparticles have also been described to release silver ions intimate the bacterial cells, additional improving their bacterial activity [44]. In our study, silver nanoparticle with the addition of curcumin-assisted chitosan nanocomposite (SCCN) by green synthesis presented pronounced antibacterial activity against gram-positive bacteria when compared to gram-negative. Combining nanocomposite that of silver ions is helpful to reduce the dose need to be directed for total microbial reduction.

#### 3.6.1. Growth Kinetic Assay of Pseudomonas aeruginosa

Figure 8 shows that the image of growth kinetics of *Pseudomonas aeruginosa.* Growth kinetics refers to the proportion at which the number of individual cells of active biomass changes in a defined system. The dose dependent activity of silver nanoparticles and its based nanocomposite was studied against the bacterial strain *Pseudomonas aeroginosa*. The growth was monitored at different time intervals by measuring absorbance at 620 nm using microplate reader. The extend of growth inhibition on SCCN by *Pongamia pinnata* was found by 56.9% at 20 *μ*g/mL, 67.29% at 40 *μ*g/mL,79.6% at 80 *μ*g/mL, 84.9% at 160 *μ*g/mL, and 90.3% at 320 *μ*g/mL, respectively. The concentration above 320 *μ*g/mL was found to be inhibitory more than 90.3% of the bacteria. When the concentration increased, the inhibition level of bacteria also increased. In this growth inhibition assay, control value is stable for percentage calculation.

The article "Curcumin-Chitosan Nanocomposite Formulation Containing Pongamia pinnata-Mediated Silver Nanoparticles, Wound Pathogen Control, and Anti-Inflammatory Potential" was retracted in 2024. Reasons: signs of a paper mill; compromised peer review; unreliable results or conclusions.

#### 3.6.2. Growth Kinetic Assay of Staphylococcus aureus

Figure 9 shows the image of growth kinetic assay of *Staphylococcus aureus*. Growth kinetics is an autocatalytic reaction, which implies that the rate of growth is directly proportional to the concentration of cell. The dose reliant to the effect of silver nanoparticle with the addition of curcumin-assisted chitosan nanocomposite (SCCN) was studied against the bacteria *Staphylococcus aureus*. The growth was monitored at different time intervals by measuring absorbance at 620 nm using microplate reader. The extend of growth inhibition on silver nanoparticle with the addition of curcumin-assisted chitosan nanocomposite (SCCN) by *Pongamia pinnata* was found by 14.0% at 20 *μ*g/mL, 30.9% at 40 *μ*g/mL, 48.4% at 80 *μ*g/mL, 60.9% at 160 *μ*g/mL, and 92.1% at 320 *μ*g/mL, respectively. The concentration above 320 *μ*g/mL was found to be inhibitory more than 92.1% of the bacteria. When the concentration increased, the inhibition level of bacteria also increased. In this growth inhibition assay, control value is stable for percentage calculation.

## 4. Conclusion

It is found that silver nanoparticles with the addition of curcumin-assisted chitosan nanocomposite (SCCN) have a significant function and strong antibacterial, anti-inflammatory, and cytotoxicity actions, hence inhibiting bacterial growth at low drug concentrations. This study proposes an ecofriendly biocompatible strategy for the creation of silver nanoparticles using green synthesis techniques based on the biocompound curcumin and the biopolymer chitosan, both of which are reducing and stabilizing agents. The experiments that ensured the creation of nanoparticles included UV visible spectroscopy, TEM, and SAED. The UV region of silver nanoparticles with the addition of curcumin-assisted chitosan nanocomposite (SCCN) added showed a peak of absorption at 350 nm. The silver nanoparticles with the addition of curcumin-assisted chitosan nanocomposite (SCCN) have a spherical form with a range of 200 nm, according to TEM. SAED demonstrates the face-centered cubic structure of silver nanoparticles with the addition of curcumin-assisted chitosan nanocomposite (SCCN).

The article "Curcumin-Chitosan Nanocomposite Formulation Containing Pongamia pinnata-Mediated Silver Nanoparticles, Wound Pathogen Control, and Anti-Inflammatory Potential" was retracted in 2024. Reasons: signs of a paper mill; compromised peer review; unreliable results or conclusions.

## Figures and Tables

**Figure 1:** UV image of Ag NPs, chitosan, and silver nanoparticle with the addition of curcumin-assisted chitosan nanocomposite (SCCN).

**Figure 2:** SEAD image of silver nanoparticle with the addition of curcumin-assisted chitosan nanocomposite (SCCN).

**Figure 3:** Transmission electron microscopic image of silver nanoparticles and silver nanoparticle with the addition of curcumin-assisted chitosan nanocomposite (SCCN).

**Figure 4:** Anti-inflammatory activity of silver nanoparticles, curcumin, and chitosan.

**Figure 5:** Anti-inflammatory activity of silver nanoparticles and silver nanoparticle with the addition of curcumin-assisted chitosan nanocomposite (SCCN).

**Figure 6:** Cytotoxic effect of nanoparticles and nanocomposites using brine shrimp lethality assay.

**Figure 7:** The antibacterial activity of silver nanoparticle with the addition of curcumin-assisted chitosan nanocomposite (SCCN).

**Figure 8:** Growth kinetics of *Pseudomonas aeruginosa.*

**Figure 9:** Growth kinetic assay of *Staphylococcus aureus.*

## Data Availability

The authors confirm that the data supporting the findings of this study are available within the article.
